RETRACTED

# Observation on the Curative Effect of Microsurgery in 154 Children with Strabismus and Analysis of Its Influencing Factors

**DOI:** 10.1155/2021/3597084

**Published:** 2021-10-18

**Authors:** Zhihua Zhao, Kejun Li, Qingmin Ma, Xiaobin Zhao, Zhiyang Jia

**Affiliations:** Department of Ophthalmology, Hebei General Hospital, Shijiazhuang, Hebei 050000, China

## Abstract

Strabismus is a common ophthalmic disease in the process of child body development, in which the two eyes cannot gaze at the target at the same time, and the incidence of this disease of children is higher. In children with esotropia, exotropia, and up and down strabismus and other typical symptoms, the cause is genetic, innerve, and refractive and regulated, and not receiving timely treatment may lead to stereo vision and diplopia and other phenomena, affecting their learning and life. Surgical treatment is the main treatment for strabismus at present. Traditional orthodontic surgery is performed by doctors under the naked eye, often due to improper operation or suture error and other factors, resulting in more postoperative complications, such as more tissue damage, conjunctival congestion, and muscle suture reaction, which seriously affect the clinical effect of surgical treatment. In recent years, with the continuous development of microsurgical technology, the correction of strabismus under a microscope has been widely carried out in clinic. The operation under the microscope makes the operation more delicate and accurate, overcomes the defects of traditional surgery, and highlights the advantages of minimally invasive surgery. The purpose of this study was to investigate the effect of microsurgical techniques in the treatment of strabismus in children and to analyze the factors influencing the outcome. The results showed that microsurgical strabismus correction in the treatment of strabismus children has short operation time, less intraoperative blood loss, short hospital stay, high efficiency, and less complications, which is worthy of popularization. Age, preoperative strabismus angle, refractive error, distance stereopsis injury, near stereoscopic injury, and duration of disease were all independent influencing factors of postoperative efficacy.

## 1. Introduction

Strabismus refers to the inability of both the eyes to look at the target at the same time, which is an extraocular muscle disease and can be divided into two categories: concomitant strabismus and paralytic strabismus [1, 2]. Among them, the main clinical features of concomitant strabismus are that there is no eye movement disorder, and the strabismus degree in the first eye position and the second eye position is equal. Paralytic strabismus is characterized by limited eye movement and diplopia, which can be congenital or caused by trauma or systemic diseases [3, 4]. The incidence of strabismus in preschool children can reach 2∼5%, which can seriously damage children's stereopsis, bring adverse effects to children's future study and life, and also bring serious adverse effects to children's mental health development [5, 6]. The treatment of strabismus includes nonsurgical treatment and surgical treatment. Nonoperative treatment includes follow-up observation, orthophoto training, wearing prism, and correcting with negative spherical lens. It is generally believed that nonsurgical treatment cannot effectively improve strabismus, and surgical treatment is still needed in the end. Surgical correction is an effective method to treat strabismus. Successful surgical correction of children's eye position can prevent the deepening of retinal inhibition scotoma, thus improving the binocular monocular function of children with strabismus [7, 8]. In the past, strabismus correction operations were mostly carried out under direct vision, which can achieve good results, but it is easy to cause damage to surrounding tissues, with more bleeding and more postoperative complications. Therefore, choosing an operation with less trauma, less pain, and less postoperative complications, and without affecting the aesthetic appearance of children, has become the goal pursued by children's families and doctors [9, 10]. In recent years, with the continuous progress of science and technology, microsurgery has been widely used in clinic. It is reported that microsurgical treatment for children with strabismus not only changes the appearance of strabismus and achieves the cosmetic effect but also heals quickly and has fewer complications, thus improving the quality of ophthalmic technology [11, 12]. The purpose of this study is to explore the curative effect of the microsurgical technique on strabismus in children and to analyze the related factors affecting the curative effect of children. Specific reports are as follows.

RETRACTED

## 2. Materials and Methods

### 2.1. Patients

154 children with strabismus treated in our hospital from June 2018 to March 2021 were selected as research objects. Among them, there were 86 males and 68 females with an average age of (4.96 ± 1.79) years, ranging from 1 to 9 years. There were 92 cases of concomitant strabismus and 62 cases of paralytic strabismus. The mean strabismus degree was (34.56 ± 9.82)°. Inclusion criteria: after admission, the patient's far and near visual acuity and corrected visual acuity were examined in detail. To high myopia and astigmatism and adolescent patients, refractive examination must be undertaken after dilating pupil, all in accordance with strabismus diagnostic standard; all patients underwent strabismus surgery in our hospital; age <10 years; and complete clinical data. Exclusion criteria: glaucoma, corneal diseases, and other eye diseases; patients with coagulation dysfunction; complicated with severe liver and kidney dysfunction; unable to cooperate with the inspection and timely review; and dysfunction of the lacrimal gland. All patients were randomly divided into the control group and observation group, with 77 cases in each group. There was no statistically significant difference between the two groups of general information (*P* < 0.05), and they were comparable, as shown in Table 1.

### 2.2. Treatment Methods

All patients were examined with naked eye vision, corrected vision, and eye movement before operation, and routine examination of the anterior segment and fundus was performed to exclude other organic eye diseases.

In both groups, 1.5 g/L Alcain eye drops were used for surface anesthesia, which were dripped into the conjunctival sac at a rate of 3 drops/time, once/4 min, and then operated after 3 times. In the control group, strabismus correction under direct vision was adopted: the conjunctiva was cut at the fornix, the extraocular muscles were separated while the muscle sheath was intact, the required muscle length was measured, and then, the extraocular muscles were retreated and sutured.

The observation group was treated with microsurgical strabismus correction: the magnification of the microscope was 6∼10 times, and the choice of the operation mode was determined according to the degree of strabismus of children. During the operation, the rectus muscle was fully exposed, the intermuscular membrane was cut off, the integrity of the muscle sheath was ensured, a conjunctival incision was made, the extraocular muscle was hooked out, the muscle length was measured, and then, the extraocular muscle was amputated. We make an incision in the conjunctiva of the infratemporal fornix, turn over the bulbar conjunctiva to hook up the inferior oblique muscle, clamp it with the hemostatic forceps, cut it off, and sew the muscle with absorbable suture. After operation, both groups of children were given functional training, such as external function and collective function, twice a day.

### 2.3. Observation Indicators

The operation time, blood loss, hospital stay, and visual acuity recovery were recorded in both groups. All the children were followed up for 6 weeks after operation, and the curative effects of the two groups were evaluated. The evaluation criteria were as follows: cure: after surgery and rehabilitation training, the strabismus of the children was ≤5°; effective: after surgery and rehabilitation training, the strabismus degree of children is between 5° and 10°; invalid: after surgery and rehabilitation training, the strabismus degree of the child is ≥10°; and effective rate = (cured + effective) cases/total cases × 100%. Complications such as muscle slippage, conjunctival congestion, and scar formation were recorded during follow-up. According to the curative effect, the children were divided into two subgroups: the effective group (cured + effective) and ineffective group. The clinical data of sex, age, strabismus type, strabismus angle before operation, refractive error, distance stereopsis injury, family history, amblyopia, and duration of disease were recorded. The related factors affecting the curative effect of children were analyzed by univariate and multivariate analysis.

RETRACTED

### 2.4. Statistical Methods

The results of this experiment were statistically analyzed by SPSS 20.0 (SPSS Co., Ltd., Chicago, USA). Count data were expressed by (rate), and the chi-square test was used for their comparison between groups. Measurement data were expressed by (mean ± standard deviation), and the *t*-test was used for their comparison between groups. Multivariate analysis adopts the multiple logistic regression model. *P* < 0.05 indicates that the difference is statistically significant.

## 3. Results

### 3.1. Comparison of Operation Time, Blood Loss, Hospital Stay, and Visual Acuity Recovery between the Two Groups

The operation time, blood loss, and hospital stay in the observation group were lower than those in the control group, and the visual acuity recovery was higher than that in the control group (*P* < 0.05), as shown in Figure 1.

### 3.2. Comparison of Curative Effects between the Two Groups

In the control group, 22 cases were cured, 44 cases were effective, 11 cases were ineffective, and the effective rate was 85.71% (66/77). In the observation group, 28 cases were cured, 46 cases were effective, 3 cases were ineffective, and the effective rate was 96.10% (74/77). The effective rate of the observation group was higher than that of the control group (*P* < 0.05), as shown in Figure 2.

### 3.3. Comparison of Complications between the Two Groups

During the follow-up, 2 cases of muscle slippage, 3 cases of conjunctival congestion, and 4 cases of scar formation occurred in the control group, and the total incidence of complication was 11.69% (9/77). In the observation group, 1 case of muscle slippage and 1 case of conjunctival congestion occurred, and the total incidence of complications was 2.60% (2/77). The total incidence of complications in the observation group was lower than that in the control group (*P* < 0.05), as shown in Figure 3.

RETRACTED

### 3.4. Univariate Analysis of Influencing the Curative Effect of Children

Univariate analysis showed that age, preoperative strabismus angle, refractive error, distance stereopsis injury, near stereoscopic injury, family history, amblyopia, and duration of disease were all related to the curative effect of children (*P* < 0.05), as shown in Table 2.

### 3.5. Multivariate Analysis of Influencing the Curative Effect of Children

Multivariate logistic analysis showed that age, preoperative strabismus angle, refractive error, distance stereopsis injury, near stereoscopic injury, and duration of disease were all independent influencing factors of curative effect (*P* < 0.05), as shown in Tables 3∼4.

## 4. Discussion

Strabismus is a common eye disease in children's physical development, which means that both the eyes cannot focus on the target at the same time, and the incidence in children is high. Children show typical symptoms such as esotropia, exotropia, and strabismus up and down, and the causes are heredity, innervation, refraction and adjustment, etc. Failure to receive timely treatment may lead to stereoscopic vision weakening and diplopia, which will affect their study and life [13, 14]. At present, the main treatment for strabismus is surgery. Strabismus correction surgery can restore the balance of extraocular muscle strength by weakening the muscles with excessive contraction and strengthening the muscles with insufficient contraction [15, 16]. After surgical treatment, the patient can get the ideal first eye position, change the strabismus appearance, achieve the cosmetic effect, and further improve the quality of life. The strabismus correction surgery requires the operator to be familiar with the relevant anatomical knowledge of the eyeball. Traditional correction surgery is carried out by doctors under the naked eye, which easily leads to many postoperative complications, such as more tissue damage, conjunctival congestion, and muscle suture reaction, which seriously affect the clinical effect of surgical treatment [17, 18]. In recent years, with the continuous development of microsurgery technology, strabismus correction under a microscope has been widely carried out in clinic. Operation under the microscope makes the operation more precise and accurate, overcomes the defects of traditional operation, and highlights the advantages of minimally invasive surgery [19, 20].

The results showed that the operation time, blood loss, and hospital stay in the observation group were lower than those in the control group, the effective rate was higher than that in the control group, and the visual acuity recovery was higher than that in the control group. Compared with strabismus correction under direct vision, microsurgical strabismus correction has the advantages of shorter operation time, less blood loss, shorter hospitalization time, and higher effective rate. The reasons are as follows: the microsurgical strabismus correction can accurately and regularly share the depth of the position passing through the sclera, avoid the phenomenon of muscle slippage, ensure that the suture is right-angled and fixed when passing through the sclera vertically, and prevent the posture change from affecting the operation process; meanwhile, we adjust the magnification and brightness of the microscope based on the actual condition of the child, so as to clearly display the anatomical level of the eye, prevent the damage to the integrity of the fascia sac during the operation, reduce the incidence of complications such as scar hyperplasia and conjunctival cyst, and ensure the integrity of the muscle sheath and tendon. The results of this study showed that the total incidence of complications in the observation group was lower than that in the control group. It shows that microsurgical strabismus correction is safe and has fewer complications. The reason is that the important blood supply source of the anterior segment of the eye is the anterior ciliary artery, which is cut off at the same time when the rectus muscles are cut off by surgery under direct vision, and 2∼3 rectus muscles are treated during operation, which may lead to complications such as anterior uveitis and anterior segment ischemia after operation. Therefore, the purpose of blood vessel separation and preservation can be achieved by microscope operation, especially for complicated strabismus and strabismus with arteriosclerosis, and the anterior ciliary artery can be preserved after precise separation. Only 3∼4 muscles need to be treated once after the muscle fibers are severed, which avoids reoperation, relieves the family economic burden of children, improves the quality of ophthalmic surgery, and reduces the complication rate of surgery under direct vision [21, 22].

RETRACTED

Univariate analysis in this study showed that age, preoperative strabismus angle, refractive error, distance stereopsis injury, near stereoscopic injury, family history, amblyopia, and duration of disease were all related to the curative effect of children. Multivariate logistic analysis showed that age, preoperative strabismus angle, refractive error, distance stereopsis injury, near stereoscopic injury, and duration of disease were all independent influencing factors of curative effect. The reasons are as follows: human stereoscopic vision mainly appears in 3∼4 months after birth, basically matures at 3∼4 years of age, and ends at 9 years of age. According to the development process of human stereoscopic vision, it can be seen that it is the best treatment opportunity for strabismus children to receive corresponding surgical correction treatment at 3∼5 years of age, which is more conducive to the recovery of children's stereoscopic vision after surgical correction [23, 24]. On the other hand, if the best treatment time is missed, with the increase of the age and duration of strabismus children, pathological changes such as macula and abnormal retinal correspondence will easily appear, which will directly affect the recovery of stereoscopic vision after operation. Therefore, it is very important to find strabismus in children as early as possible and give timely treatment. The larger the oblique angle is, the more serious the damage to the third-level function of the same vision machine is. The more unfavorable it is to the reconstruction of binocular visual function after operation. Children with strabismus need fusion reserve to control eye position deviation. When eye position deviation is small and can be controlled by motion fusion, they show good binocular monocular function. The larger the squint angle, the greater the fusion force needed. Once the compensation range of motor fusion is exceeded, obvious eye position deviation will appear, which will damage binocular visual function. The longer the course of the disease, the greater the hindrance to stereoscopic vision development, which is not conducive to postoperative recovery [25, 26]. Human stereoscopic vision mainly appears in 3-4 months after birth and develops basically maturely at the age of 3-4. The development of stereoscopic vision ends at the age of 9. According to the development process of human stereoscopic vision, it can be seen that the optimal treatment timing is for children with strabismus to receive corresponding surgical correction at the age of 3–5. It is more conducive to the recovery of stereoscopic vision of children after surgical correction. Therefore, surgical treatment should be carried out as far as possible before stereoscopic injury in children, which is beneficial to improve the visual recovery of children.

## 5. Conclusions

Microsurgical strabismus correction for children with strabismus has the advantages of short operation time, less blood loss, short hospital stay, high effective rate, and few complications, which is worth popularizing. Age, preoperative strabismus angle, refractive error, distance stereopsis injury, near stereoscopic injury, and duration of disease are all independent influencing factors of the postoperative curative effect of strabismus children.

RETRACTED

## Figures and Tables

**Figure 1:** Comparison of operation time, blood loss, hospital stay, and visual acuity recovery between the two groups. Note: compared with the control group, ^*∗*^*P* < 0.05.

**Figure 2:** Comparison of curative effects between the two groups. Note: compared with the control group, ^*∗*^*P* < 0.05.

**Figure 3:** Comparison of complications between the two groups. Note: compared with the control group, ^*∗*^*P* < 0.05.

**Table 1:** Comparison of general data between the two groups.

Groups	*n*	Age (years)	Gender		Strabismus degree (°)
			Male	Female	
Control group	77	4.89 ± 1.92	46	31	34.47 ± 9.91
Observation group	77	5.03 ± 1.70	40	37	34.65 ± 9.65
*t*/*χ*^2^		0.479	0.948		0.114
*P*		0.633	0.331		0.909

**Table 2:** Univariate analysis of influencing the curative effect of children.

Factor	*n*	Effective group (*n* = 140)	Ineffective group (*n* = 14)	*t*/*χ*^2^	*P*
Gender				1.517	0.218
Male	86	76 (54.29)	10 (71.43)		
Female	68	64 (45.71)	4 (28.57)		

Age (years)	154	4.81 ± 1.58	6.46 ± 1.79	3.681	0.001

Strabismus type				0.132	0.716
Comorbicular strabismus	92	83 (59.29)	9 (64.29)		
Paralytic strabismus	62	57 (40.71)	5 (35.71)		

Preoperative strabismus angle (°)				4.129	0.042
≥30	93	81 (57.86)	12 (85.71)		
<30	61	59 (42.14)	2 (14.29)		

Refractive error				7.404	0.007
Yes	26	20 (14.29)	6 (42.86)		
No	128	120 (85.71)	8 (57.14)		

Distant stereopsis injury				10.481	0.001
Yes	28	21 (15.00)	7 (50.00)		
No	126	119 (85.00)	7 (50.00)		

Near stereoscopic injury				7.404	0.007
Yes	26	20 (14.29)	6 (42.86)		
No	128	120 (85.71)	8 (57.14)		

Family medical history				6.212	0.013
Yes	15	11 (7.86)	4 (28.57)		
No	139	129 (92.14)	10 (71.43)		

Complicated with amblyopia				5.365	0.021
Yes	30	24 (17.14)	6 (42.86)		
No	124	116 (82.86)	8 (57.14)		

Duration of disease (years)				12.697	<0.001
≤1	108	104 (74.29)	4 (28.57)		
>1	46	36 (25.71)	10 (71.43)		

**Table 3:** Assignment for multivariate analysis of factors.

Factors	Variable	Assignment
Age	X1	Continuous variable
Preoperative strabismus angle	X2	<30 = 0, ≥30 = 1
Refractive error	X3	No = 0, Yes = 1
Distant stereopsis injury	X4	No = 0, Yes = 1
Near stereoscopic injury	X5	No = 0, Yes = 1
Family medical history	X6	No = 0, Yes = 1
Complicated with amblyopia	X7	No = 0, Yes = 1
Duration of disease	X8	≤1 = 0, >1 = 1

**Table 4:** Multivariate analysis of influencing the curative effect of children.

Variables	*B*	S.E	Walds	*P*	OR	95% CI
Age	0.652	0.167	8.694	<0.001	1.919	1.415∼2.564
Preoperative strabismus angle	1.293	0.368	10.154	<0.001	3.644	1.518∼7.647
Refractive error	0.342	1.358	4.216	0.041	1.408	1.089∼1.965
Distant stereopsis injury	0.386	1.402	4.961	0.038	1.471	1.105∼1.894
Near stereoscopic injury	0.396	1.538	5.169	0.035	1.486	1.052∼2.041
Family medical history	2.965	3.061	0.375	0.869	19.395	0.068∼60.452
Complicated with amblyopia	1.029	2.105	1.496	0.185	2.798	0.052∼14.395
Duration of disease	1.072	0.325	9.164	<0.001	2.921	1.564∼5.381

RETRACTED

## Data Availability

The data can be obtained from the author upon reasonable request.
